The article "Analysis of Causes and Results of Fetal Growth in Utero Caused by Genetic Factors Detected by Ultrasound" was retracted in 2023. Reasons: suspected computer-generated content; unreliable results or conclusions; concerns about the data; concerns about the results or conclusions.

# Analysis of Causes and Results of Fetal Growth in Utero Caused by Genetic Factors Detected by Ultrasound

**DOI:** 10.1155/2022/3703132

**Published:** 2022-08-31

**Authors:** Mei Yu, Ying Liu, Liya Wang

**Affiliations:** ^1^Prenatal Diagnosis Center, The Fourth Hospital of Shijiazhuang (The Obstetrics and Gynecology Hospital of Hebei Medical University), Shijiazhuang, Hebei, China; ^2^Obstetrical Department VIII, The Fourth Hospital of Shijiazhaung (The Obstetrics and Gynecology Hospital of Hebei Medical University), Shijiazhuang, Hebei, China; ^3^Neonatal Surgery, The Fourth Hospital of Shijiazhuang (The Obstetrics and Gynecology Hospital of Hebei Medical University), Shijiazhuang, Hebei, China

## Abstract

In order to investigate the value of the ultrasonic monitoring of maternal and fetal vascular parameters, serum vitamin D, and placental growth factor (PLGF) in predicting fetal growth restriction (FGR), a method of ultrasonic detection of genetic factors causing fetal growth in utero was proposed. 125 pregnant women with FGR diagnosed in our hospital from June 2018 to June 2021 (the FGR group) and 125 pregnant women with a normal prenatal examination (the control group) were collected retrospectively. The systolic/diastolic blood flow ratio (S/D), pulsatile index (PI), and resistance index (RI) of the fetal umbilical artery (UA), middle cerebral artery (MCA), and maternal uterine artery (UtA) were monitored by ultrasound at 20 to 24 weeks of gestation, and the levels of serum vitamin D and PLGF were detected. The receiver operating characteristic curve (ROC curve) was used to evaluate the predictive value of FGR. The results showed that the S/D, PI, and RI of UA in the FGR group were higher than those in the control group, the areas under the curve (AUC) were 0.866, 0.817, and 0.849, and the sensitivity and specificity were (72.8%, 91.2%), (50.4%, 100%), and (72.8%, 91.2%), respectively. The S/D, PI, and RI of MCA were lower than those of the control group. The AUC was 0.882, 0.869, and 0.834, respectively; the sensitivity and specificity were (92.0%, 74.4%), (88.8%, 81.6%), and (90.4%, 72%), respectively. The S/D, PI, and RI of UtA were higher than those of the control group; the AUC was 0.768, 0.729, and 0.732; the sensitivity and specificity were (91.2%, 52%), (48%, 90.4%), and (48.8%, 90.4%), respectively. The serum levels of vitamin D and PLGF were lower than those of the control group (AUC 0.784 and 0.807), and the sensitivity and specificity were (54.4%, 91.2%) and (99.2%, 52%), respectively. It was concluded that the ultrasound monitoring of UA, MCA, and UtA in pregnant women in the middle of pregnancy and detection of serum vitamin D and PLGF levels had a certain predictive value for FGR. Moreover, the comprehensive evaluation could reduce the occurrence of FGR in high-risk pregnant women.

The article "Analysis of Causes and Results of Fetal Growth in Utero Caused by Genetic Factors Detected by Ultrasound" was retracted in 2023. Reasons: suspected computer-generated content; unreliable results or conclusions; concerns about the data; concerns about the results or conclusions.

## 1. Introduction

Fetal growth restriction (FGR), also known as intrauterine growth retardation (IUGR), refers to the fetus's inability to reach its proper growth potential in the womb due to various adverse reasons. The results show that the fetal weight is lower than the 10th percentile of the fetal weight at the same gestational age or 2 standard deviations lower than the average fetal weight at the same gestational age, the fetal weight is lower than the 3rd percentile, and the fetus with abnormal Doppler flow under the color Doppler ultrasound is classified as having severe FGR. Generally, the weight of a fetus delivered at 37 weeks of gestation should be more than 2500 g. If less than 2500 g, it is called low birth weight [1]. According to the epidemiological investigation, the incidence of FGR ranges from 2.75% to 15.53%, among which the average incidence in developing countries is 11.2%, 6 times higher than that in developed countries. According to statistics, the incidence of FGR in China is about 6.39%. It is listed as one of the most important common obstetric complications, which increases the risk of fetal and neonatal morbidity and mortality significantly during the perinatal period. The perinatal mortality of children with FGR is 4∼6 times that of normal fetuses, accounting for 42.3% of the death causes of perinatal children in China, which is the second influential factor leading to neonatal deaths [2]. Initially, FGR is simply divided into symmetrical and nonsymmetrical types. With the deepening of the understanding of FGR in recent years, domestic and foreign experts agree that it can be divided into three types, namely, endogenous symmetry FGR, external asymmetrical FGR, and external symmetrical FGR , based on mainly the time of occurrence, fetal weight, and etiology. Endogenous symmetry, also known as primary FGR, accounts for 18.18% of all FGR. Due to the harmful factors acting on the embryo in the early stages of pregnancy, the fetal weight, body length, and the head circumference (HC) are restricted, and head circumference and abdominal circumference (AC) are small, so it is called a symmetry type. The main harmful factors are genetic or chromosomal diseases, exposure of pregnant women to radioactive substances, viral infections, and so on. Exogenous asymmetric FGR accounts for about 67.27%, mainly due to the effects of harmful factors in late pregnancy. The fetal head circumference and body length develop normally, but its weight is low. The common harmful factors include hypertensive disorders complicating pregnancy (HDCP), diabetes mellitus (GDM), chronic nephritis, overdue pregnancy, etc. The pathological mechanism is mainly placental dysfunction and uterine-placental insufficiency. This results in the lack of nutrients needed for fetal development, which is manifested as malnutrition [3, 4]. The proportion of external symmetrical FGR is 14.55%, and adverse factors exist during the whole pregnancy because of the lack of important nutrients such as amino acids and folic acid. The fetal performance is similar to that of internal symmetrical FGR, with smaller head circumference, body weight, and body length. FGR can not only lead to adverse outcomes for the perinatal fetus and newborn but also have a profound long-term impact on children. Although most children with FGR have caught up with their peers in terms of height and weight at 6 months or 1 year old, respectively, children with FGR are at higher risk of developing mild cognitive impairment, ADHD, and attention deficiency in childhood. With the development of maternal and fetal medicine in recent years, more and more experts are committed to studying how to reduce the occurrence of related diseases in adulthood by avoiding harmful factors for the fetus during pregnancy. FGR has become one of the research hotspots due to the complexity of its causes and far-reaching influence See Figure 1:

The article "Analysis of Causes and Results of Fetal Growth in Utero Caused by Genetic Factors Detected by Ultrasound" was retracted in 2023. Reasons: suspected computer-generated content; unreliable results or conclusions; concerns about the data; concerns about the results or conclusions.

## 2. Literature Review

By the clinical measurement of uterine height and abdominal circumference, the gestational age of the fetus can be roughly estimated and the fetal growth screening is performed. But the accuracy is affected by maternal obesity, pregnancy times, and uterine fibroids. The ultrasound examination is a good means for screening, diagnosis, and monitoring of FGR. However, there is still no international agreement on the relevant definition and ultrasound diagnostic standard of FGR, and there are also controversies about the clinical application of prenatal ultrasound monitoring indicators. It is still difficult to distinguish FGR from healthy small for gestational age (SGA). The research by Smith, showed that the existing customized and population-based growth curves could identify SGA with adverse outcome risks, but no direct comparison was made [5]. Chen, found that among fetuses with an estimated body mass less than the 10th percentile, the slow growth rate during the middle and late pregnancy was associated with the poor pregnancy prognosis [6]. The research by Schoots showed that the slow growth rate (estimated body mass over 30% on the growth curve compared with previous growth) was associated with the abnormal cerebroplacental blood flow ratio (the ratio of the pulsatile index of the middle cerebral artery to the umbilical artery), but with low predictive value. Recent retrospective research showed that the slow fetal growth rate was associated with the abnormal blood flow spectrum of the umbilical artery and middle cerebral artery but was not an independent influencing factor of adverse pregnancy outcomes [7]. The research by Chen showed that the late FGR with the abnormal uterine artery blood flow spectrum had a two-fold increased risk of abnormal cerebral blood flow before the delivery [8]. In a randomized controlled study involving 11667 pregnant women, Somjid found that in the general population, routine midpregnancy screening of the uterine artery blood flow spectrum was about 60% sensitive to finding placental insufficiency, but this screening method did not improve the perinatal mortality and morbidity of pregnant women and neonates. Although the prediction value of the uterine artery blood flow spectrum was limited, it was very beneficial for identifying preeclampsia, a high-risk factor for FGR. So, some national guidelines suggested monitoring the uterine artery blood flow spectrum for high-risk groups [9]. Macdonald's meta-analysis showed that oligohydramnios were associated with the Apgar score after birth of FGR, but not with perinatal mortality and acidosis. Currently, taking the amniotic fluid volume as a prognostic monitoring indicator of FGR is not sufficient [10].

The article "Analysis of Causes and Results of Fetal Growth in Utero Caused by Genetic Factors Detected by Ultrasound" was retracted in 2023. Reasons: suspected computer-generated content; unreliable results or conclusions; concerns about the data; concerns about the results or conclusions.

In the research, UA, MCA, UtA, and other vascular parameters, as well as vitamin D and PLGF levels, were analyzed retrospectively in pregnant women with FGR, so as to explore the predictive value of each indicator for FGR and provide a reference for the early diagnosis of FGR.

## 3. Research Methods

### 3.1. Data and Methods

#### 3.1.1. General Information

The clinical data of 125 pregnant women with FGR diagnosed in a hospital from June 2018 to June 2021 were selected (the FGR group). The inclusion criteria are as follows: (1) meeting the diagnostic criteria of FGR; (2) single child; (3) complete medical records; and (4) signing the informed consent. The exclusion criteria are as follows: (1) complicated by pregnancy complications; (2) chromosomal abnormalities; (3) assisted reproductive pregnancy; (4) abnormal coagulation function in pregnant women; (5) combined with underlying diseases; and (6) intrauterine infection during pregnancy. 125 normal pregnant women (the control group) received prenatal examinations during the same period. This research was approved by the Ethics Committee of our hospital [11].

#### 3.1.2. Ultrasound Examination

All pregnant women underwent the ultrasound examination at 20–24 weeks of gestation. The color ultrasound diagnostic instrument (GE VolusonE8) with a protruding array probe frequency of 3.5–5.0 MHz was used to check the growth of the fetal head circumference, abdominal circumference, biparietal diameter, femoral diameter, humeral diameter, amniotic fluid volume, and placenta [12]. UA, MCA, and UtA blood flow parameters were measured according to the guidelines of the International Society of Obstetrical Ultrasound. End systolic peak/end diastolic peak (S/D), venous pulse index (PI), and resistance index (RI) were monitored and averaged for three times.

The article "Analysis of Causes and Results of Fetal Growth in Utero Caused by Genetic Factors Detected by Ultrasound" was retracted in 2023. Reasons: suspected computer-generated content; unreliable results or conclusions; concerns about the data; concerns about the results or conclusions.

#### 3.1.3. Laboratory Examination

Serum vitamin D and PLGF levels were detected by the high-performance liquid chromatography-tandem mass spectrometry (HPLC) method and the enzyme-linked immunosorbent assay (ELISA) method.

#### 3.1.4. Statistical Methods

SPSS22.0 was used to analyze the data. Count data (%) were performed by *χ*^2^ test. The measurement data conforming to a normal distribution ($\bar{x}\pm s$) were tested by an independent sample *t* test. The predictive value was evaluated by the receiver operating characteristic curve (ROC) [13]. *P* < 0.05 means the difference is statistically significant.

*t* test, also known as a student's *t* test, is mainly used for normal distribution data with a small sample size (e.g. *n* < 30) and unknown population standard deviation *σ*. *t* test is used to test the degree of difference between the two mean values of a small sample. It uses *t* distribution theory to infer the probability of difference, so as to determine whether the difference between two means is significant. It mainly includes three methods: single sample *t* test, paired sample *t* test and two independent samples *t* test. The basic idea of paired sample *t* test is to assume that population *X*_1_ follows a normal distribution *N*(*μ*_1_, *σ*_12_), and population *X*_2_ follows a normal distribution *N*(*μ*_2_, *σ*_22_). Samples (*x*_11_, *x*_12_,…, *x*_1*n*_) and (*x*_21_, *x*_22_,…, *x*_2*n*_) are extracted from these two populations, respectively, and the two samples are paired with each other. Whether *μ*_1_ and *μ*_2_ are significantly different needs to be tested. The specific steps are as follows:

(1) Introducing variables Introduce a new random variable *Y*=*X*_1_ − *X*_2_, corresponding to sample value (*y*_1_, *y*_2_,…, *y*_*n*_), *y*_*i*_=*x*_1*i*_ − *x*_2*i*_(*i*=1,2,…, *n*).
(2) Establishing hypothesis as shown in the following formula:
  (1) $$\begin{array}{c} H_{0}:\mu_{Y}=0\text{.} \end{array}$$
(3) The calculation formula and significance are shown in formula (2).
  (2) $$\begin{array}{c} t=\frac{\bar{y}}{S_{y}/\sqrt{n}}\text{.} \end{array}$$

In formula (2), $\bar{y}=\sum_{i=1}^{n}\;y_{i}/n$ is the average of the difference values of paired samples; $S_{y}=\sqrt{\sum_{i=1}^{n}\;{\left(y_{i}-\bar{y}\right)}^{2}/n-1}$ is the standard deviation of the difference of paired samples; and *n* is the number of paired samples.

The article "Analysis of Causes and Results of Fetal Growth in Utero Caused by Genetic Factors Detected by Ultrasound" was retracted in 2023. Reasons: suspected computer-generated content; unreliable results or conclusions; concerns about the data; concerns about the results or conclusions.

The statistic *t* follows a *t* distribution with *n* − 1 degree of freedom under the true null hypothesis (*μ*_*Y*_=0).

## 4. Analysis of Results

### 4.1. Results

#### 4.1.1. General Clinical Data

The FGR group has patients who are (29.6 ± 3.3) years old (20–38 years old), with (1.3 ± 0.5) pregnancies (1–4 times), 69 primiparas, and 56 paras [14, 15]. Patients in the control group are (30.5 ± 3.5) years old (21–39 years old), pregnant times (1.2 ± 0.4) (1–4 times), 67 primiparas, and 58 parturients. There is no difference between the two groups (*P* > 0.05).

#### 4.1.2. Comparison of Vascular Ultrasound Parameters between the Two Groups

The S/D, PI, and RI of UA in the FGR group are higher than those in control group, the S/D, PI and RI of MCA are lower than those in the control group, and the S/D, PI and RI of UtA are higher than those in the control group (*P* < 0.05). See Table 1 to Table 3.

#### 4.1.3. Serum Vitamin D Level

Serum vitamin D in the FGR group (24.15 ± 8.51 nmol/L) is lower than that in the control group (35.68 ± 10.62 nmol/L), and PLGF level (276.98 ± 80.46pg/ml) is higher than that in the control group (405.65 ± 93.54pg/ml) (*P* < 0.05). See Table 2.

#### 4.1.4. Using Ultrasound Parameters and Serum Indexes to Predict FGR

The ROC curve analysis shows that UA-S/D, UA-PI, UA-RI, MAC-S/D, MAC-PI, MAC-RI, UTA-S/D, UTA-PI, UTA-RI, vitamin D, and PLGF are all valuable in predicting FGR [16]. See Table 4 and Figure 2.

### 4.2. Discussions

FGR is not only prone to an adverse fetal pregnancy outcome but also leads to increased risks of postnatal intellectual development and cardiovascular diseases. The early prediction of the risk of FGR is of great significance for the healthy growth of fetuses. Uterine height measurement can judge whether the weight of the fetus is normal, but it is easy to confuse it with a child of less than gestational age, resulting in false positives. Therefore, a more appropriate examination method should be found [17].

Placental blood vessels are the basis for fetuses to obtain oxygen and nutrients. The vascular endothelial cell growth factor (VEGF) family can regulate the functions of placental trophoblast cells and endothelial cells. It plays a key role in placental angiogenesis and promotes the fetal growth and development. VEGF-A and PLGF are members of the VEGF family. The placental blood vessels begin to form in the early stage of pregnancy, when VEGF-A plays a major role. In the second trimester, new blood vessels are formed through the proliferation and budding of existing capillaries, and the capillary density increases. At this time, PLGF appears in the fetal disc in a large amount, while the expression of VEGF-A decreases [18, 19]. The results of this research show that the PLGF expression level in the FGR group is lower than that in the control group in the middle of pregnancy, suggesting that the placental angiogenesis of FGR pregnant women is impaired and the fetus is unable to obtain adequate nutrition, resulting in the slow development. From the further ROC analysis, it is found that PLGF has a high predictive value, but its specificity is slightly lower, and there is a certain risk of misdiagnosis. The possible reason is that soluble vascular endothelial growth factor receptor-1 (sFlt-1), as an angiogenic inhibitor, can inhibit its activity by binding with PLGF, so that the angiogenic effect of PLGF cannot be exerted [20].

The article "Analysis of Causes and Results of Fetal Growth in Utero Caused by Genetic Factors Detected by Ultrasound" was retracted in 2023. Reasons: suspected computer-generated content; unreliable results or conclusions; concerns about the data; concerns about the results or conclusions.

Pregnant women's blood is usually in a hypercoagulable state to protect the mother and fetus from bleeding, but there is some risk of FGR. UA is the link between fetal and maternal blood circulation and can reflect the pathological changes of the placenta and the mother. With the increase in gestational age and placenta development, fetal demand for nutrients increases and UA blood flow resistance decreases and blood flow increases [21]. The results of the research show that the S/*D*, PI, and RI parameters of UA in the FGR group are higher than those in the control group, which may be related to the decrease in the number of placental villi, the lack of villi vessels, and the insufficiency of blood flow perfusion in fetuses of the FGR group. The S/D, PI, and RI parameters all have certain value in predicting FGR, but their sensitivity is slightly lower. It may be related to the fact that UA blood flow parameters of fetuses with late FGR do not change significantly in the middle of pregnancy, which leads to the inability to determine the occurrence of FGR accurately [22]. The MCA, as a branch of the internal carotid artery, is an important blood vessel of the fetal brain. When FGR occurs in the fetal brain, cerebral ischemia and hypoxia will lead to “blood redistribution” phenomenon. The blood flow of the brain will increase, while the blood flow of UA will decrease to ensure sufficient blood flow to the brain to maintain the brain development and it is the same as the research results. The results show that the S/D, PI, and RI parameters of MAC all have a certain value in predicting FGR, but the specificity is slightly lower, which may be caused by a cerebral vascular compensatory diastolic loss in severe brain hypoxia, leading to MCA abnormalities that cannot truly reflect the pathological changes of the brain, thus affecting the accuracy of FGR prediction. UtA is the direct source of maternal nutrition delivery to the fetus. Blood flow parameters of UtA reflect maternal supply capacity and placental circulation. Increased resistance to UtA affects fetal placental circulation, leading to the fetal arrest and increased risk of FGR, etc [23]. The results of the research show that the S/D, PI, and RI parameters of UtA in the FGR group are higher than those in the control group, but the sensitivity of FGR prediction is lower. Therefore, the changes in blood flow parameters in UA, MCA, and UtA should be comprehensively analyzed clinically to improve the accuracy of prediction.

The article "Analysis of Causes and Results of Fetal Growth in Utero Caused by Genetic Factors Detected by Ultrasound" was retracted in 2023. Reasons: suspected computer-generated content; unreliable results or conclusions; concerns about the data; concerns about the results or conclusions.

Vitamin D deficiency is associated with a variety of pregnancy complications, including fetal adverse pregnancy complications. The research shows that the vitamin D level in the FGR group is lower than that in the control group. Vitamin D can maintain normal pregnancy and fetal growth and development, and maternal vitamin D deficiency can lead to the occurrence of FGR [24]. It is found that vitamin D has high specificity but low sensitivity in predicting FGR, which may be related to the great fluctuation of vitamin D levels affected by various factors such as season, region, and race. Therefore, it should not be used to predict FGR alone.

## 5. Conclusions

In conclusion, the ultrasound monitoring of UA, MCA, and UtA, as well as the detection of serum vitamin D and PLGF levels in pregnant women during the second trimester of pregnancy has a certain value in predicting FGR, but there is a certain risk of missed diagnosis and misdiagnosis. Therefore, a comprehensive evaluation should be conducted for high-risk pregnant women to improve the prediction accuracy of FGR and some timely intervention measures should be taken to reduce the occurrence of FGR.

## Figures and Tables

**Figure 1:** Ultrasound tests genetic factors that cause a fetus to grow in the womb.

**Figure 2:** Vascular ultrasound parameters and sensitivity and specificity of serum vitamin D and PLGF prediction.

**Table 1:** Comparison of UA vascular parameters and ultrasonic parameters ($\bar{x}\pm s$)

Group	Cases	S/D	PI	RI
The FGR group	125	3.49 ± 0.54	1.05 ± 0.24	0.69 ± 0.11
The control group	125	2.72 ± 0.45	0.76 ± 0.16	0.56 ± 0.07
*t*		12.247	11.241	11.147
*P*		<0.001	<0.001	<0.001

**Table 2:** Comparison of MCA vascular parameters and ultrasound parameters ($\bar{x}\pm s$)

Group	Cases	S/D	PI	RI
The FGR group	125	3.93 ± 0.51	1.34 ± 0.18	0.71 ± 0.05
The control group	125	4.89 ± 0.63	1.65 ± 0.23	0.79 ± 0.07
*t*		13.242	11.867	10.398
*P*		<0.001	<0.001	<0.001

The article "Analysis of Causes and Results of Fetal Growth in Utero Caused by Genetic Factors Detected by Ultrasound" was retracted in 2023. Reasons: suspected computer-generated content; unreliable results or conclusions; concerns about the data; concerns about the results or conclusions.

**Table 3:** Comparison of UtA vascular parameters and ultrasonic parameters ($\bar{x}\pm s$)

Group	Cases	S/D	PI	RI
The FGR group	125	2.65 ± 0.53	0.98 ± 0.21	0.58 ± 0.12
The control group	125	2.06 ± 0.49	0.81 ± 0.15	0.47 ± 0.11
*t*		9.139	7.365	7.555
*P*		<0.001	<0.001	<0.001

**Table 4:** ROC analysis of vascular ultrasound parameters and serum vitamin D and PLGF in predicting FGR.

Indexes	AUC	Standard error a	Asymptotic significance level b	*95% confidence interval*		Cut-off value	Youden index	Sensitivity (%)	Specificity (%)
				Lower	Upper				
UA-S/D	0.866	0.024	0	0.819	0.912	3.185	0.640	72.8	91.2
UA-PI	0.817	0.026	0	0.767	0.868	1.065	0.504	50.4	100.0
UA-PI	0.849	0.026	0	0.797	0.900	0.635	0.640	72.8	91.2
MAC-S/D	0.882	0.022	0	0.839	0.926	4.48	0.664	92.0	74.4
MAC-PI	0.869	0.025	0		0.918	1.495	0.704	88.8	81.6
MAC-PI	0.834	0.026	0	0.782	0.885	0.755	0.624	90.4	72.0
UtA-S/D	0.768	0.029	0	0.711	0.825	2.095	0.432	91.2	82.0
UtA-PI	0.729	0.032	0	0.667	0.791	0.99	0.384	48.0	910.4
UtA-PI	0.732	0.031	0	0.670	0.793	0.595	0.392	48.8	90.4
Vitamin D	0.784	0.028	0	0.729	0.840	24.2	0.456	54.4	91.2
PLGF	0.807	0.027	0	0.755	0.860	395.705	0.512	99.2	52.0

## Data Availability

The data used to support the findings of this study are available from the corresponding author upon request.
